The article "Electrocardiogram Signal Classification in the Diagnosis of Heart Disease Based on RBF Neural Network" was published in 2022. Journal: Comput Math Methods Med.

# Electrocardiogram Signal Classification in the Diagnosis of Heart Disease Based on RBF Neural Network

**DOI:** 10.1155/2022/9251225

**Published:** 2022-01-30

**Authors:** Yan Fang, Jianshe Shi, Yifeng Huang, Taisheng Zeng, Yuguang Ye, Lianta Su, Daxin Zhu, Jianlong Huang

**Affiliations:** ^1^Faculty of Mathematics and Computer Science, Quanzhou Normal University, Quanzhou 362000, China; ^2^Fujian Provincial Key Laboratory of Data Intensive Computing, Quanzhou 362000, China; ^3^Key Laboratory of Intelligent Computing and Information Processing, Fujian Province University, Quanzhou 362000, China; ^4^Department of General Surgery, Huaqiao University Affiliated Strait Hospital, Quanzhou, Fujian 362000, China; ^5^Department of Diagnostic Radiology, Huaqiao University Affiliated Strait Hospital, Quanzhou, Fujian 362000, China

## Abstract

Heart disease is a common disease affecting human health. Electrocardiogram (ECG) classification is the most effective and direct method to detect heart disease, which is helpful to the diagnosis of most heart disease symptoms. At present, most ECG diagnosis depends on the personal judgment of medical staff, which leads to heavy burden and low efficiency of medical staff. Automatic ECG analysis technology will help the work of relevant medical staff. In this paper, we use the MIT-BIH ECG database to extract the QRS features of ECG signals by using the Pan-Tompkins algorithm. After extraction of the samples, *K*-means clustering is used to screen the samples, and then, RBF neural network is used to analyze the ECG information. The classifier trains the electrical signal features, and the classification accuracy of the final classification model can reach 98.9%. Our experiments show that this method can effectively detect the abnormality of ECG signal and implement it for the diagnosis of heart disease.

## 1. Introduction

Cardiac diseases are likely to occur in all age groups [1]. Surgery for cardiac diseases is difficult and risky. Conservative treatment is often used for nonessential cardiac diseases, which results in high recurrence probability and high diagnostic efficiency.

Electrocardiogram (ECG) detection is currently the most effective and direct way to detect ECG signals [2]. At present, the diagnosis of cardiac diseases is mainly determined by medical doctors and clinicians through manual detection and ECG analysis. The related ECG automatic analysis technology can provide effective help for the diagnosis of medical workers, which can help to improve the efficiency of diagnosis.

Based on the above problems, this paper proposes an automatic ECG analysis technology, which uses Pan-Tompkins algorithm, uses ECG data in MIT-BIH ECG database to extract the features of ECG QRS complex, and uses *K*-means clustering to filter the data after cutting the samples. Then, RBF neural network is used to train the classifier for the extracted ECG features. This method can effectively judge the abnormalities of ECG signals.

The article "Electrocardiogram Signal Classification in the Diagnosis of Heart Disease Based on RBF Neural Network" was published in 2022. Journal: Comput Math Methods Med.

ECG is a diagnostic technology that records the electrocardiography activities of the heart in a certain time unit through the chest of biological objects. It collects and records the electrodes connected to the skin of specific parts of biological objects and preserves the relevant contents in a certain form [3].

In the process of detection, several electrodes are usually placed on human limbs. These electrodes must appear in pairs, as shown in Figure 1, which is called lead. In this paper, the LL+RL electrode combination, known as one- or two-lead electrocardiograms, is used. This method is often used in one diagnosis [4]. This method coincides with the fast diagnosis direction in this paper.

Each electrode in the test result will get a corresponding ECG signal map. In this paper, the LA signal data is unified.

Although the ECG signal has a very obvious periodicity, due to the diversity of noise and random factors caused by external factors, it has become a difficult research problem for the diagnosis of ECG abnormalities [5]. Therefore, on the basis of previous studies by various scholars and experts [6], we use the compromise Pan-Tompkins paper [7] to denoise and extract features for the QRS wave group of ECG signal, use *K*-means algorithm [8] to cluster the sample wave group, select the similar ECG signal, and then use the radial basis function neural network to extract the ECG signal. The algorithm trains the feature classifier and achieves the expected results.

## 2. Methods

### 2.1. Feature Extraction

#### 2.1.1. Object Survey

To analyze ECG signal, the most necessary step is to extract its QRS wave group. The QRS complex reflects changes in depolarization potential and time of the left and right ventricles. Considering the robustness and stability, the QRS wave group is finally selected in this paper [9].

ECG signal has periodicity. Compared with other electrical signals such as brain wave and muscle wave, ECG signal belongs to a kind of wave which is easy to detect and distinguish features.

The QRS wave group is a detailed description of potential changes in ventricular depolarization (Figure 2). In the ECG signal graph, after P wave ends, Q wave enters PR interval, and then, Q wave shows a downward trend, R wave quickly goes up, and S wave immediately goes down. These three waves correspond to the connected waves, which are collectively referred to as the QRS wave group in this paper.

The article "Electrocardiogram Signal Classification in the Diagnosis of Heart Disease Based on RBF Neural Network" was published in 2022. Journal: Comput Math Methods Med.

Another very important reason for choosing the QRS wave group is that the QRS wave group is the most obvious corresponding signal in ECG signal. The correct choice of the QRS wave group is the next step to complete the selection of other signal waves.

It is obvious from Figure 2 that R wave is the narrowest and the largest of all waveforms.

T wave corresponds to the process of repolarization of human ventricular muscle; the process of cardiac depolarization corresponds to P wave, so it makes blunt circular image; PR corresponds to the process of transmission; in ideal state, there is no potential change, that is, the ECG signal is flat. The period of QT corresponds to a process of human ventricular contraction [10]. Therefore, the heart rate can be effectively detected by the change of the interval of QT. The size of the period of QT is proportional to the speed of human heart rate [11].

In normal ECG signal cycle, P wave and T wave have no obvious characteristics. If we want to distinguish them clearly, we need to detect them by the position of the QRS wave group.

#### 2.1.2. Contrastive Selection

There are many related literatures about the extraction and detection methods of the QRS wave group. The main methods are focused on wavelet transform [9], neural networks [12], classical Pan-Tompkins algorithm, and its improved algorithm [13]. The improved wavelet algorithm of notch filter [14] is added.

The accuracy of wavelet transform method is high, but the disadvantage is that its calculation steps are very tedious, so the time efficiency is not high. Secondly, the redundancy of data will increase in the process of wavelet transform. Although the neural network is a very accurate method, the performance of a neural network depends on its training model. This process is very long, and different training samples produce different training results. The above characteristics make it not suitable for practical applications. The algorithm provided in a real-time ECG filter for portable mobile medical systems [15] does not need model training, and the corresponding process of the method is more convenient and efficient than that of the wavelet transform method, which belongs to a compromise scheme.

To the best of our knowledge, this paper considers and presents the advantages and disadvantages of each method. To implement a real-time QRS detection algorithm, we adopted the RBF neural network to perform ECG classification [7].

#### 2.1.3. Extraction Process

Some mature and extremely complex algorithms are proposed in references, including low-pass filtering, high-pass filtering, differential, square, integral, adaptive threshold, and search. Based on references, this paper only gives a brief description of the implementation process.

*(1) Noise Reduction*. However, due to the different equipment and environment, different noises will be introduced in the acquisition process of electrical signals, which will inevitably affect the final judgment, so the processing of noise in ECG data is the core content of data preprocessing.

The article "Electrocardiogram Signal Classification in the Diagnosis of Heart Disease Based on RBF Neural Network" was published in 2022. Journal: Comput Math Methods Med.

High-pass filter method and low-pass filter method are used in this process. The purpose is to filter out the noise in the electrical signal, so as to improve the signal-to-noise ratio of the electrical signal.

The main noise in ECG signal is power frequency interference and baseline drift [15]. Power system and other interference signals are called power frequency interference; the frequency is generally concentrated in 50 Hz. Skin contact, human breathing, etc. will produce the so-called baseline drift; the frequency is generally concentrated in 0.05 Hz to 2 Hz. The frequency of the QRS wave group mainly concentrates on 5 Hz to 11 Hz.

Taking T as sampling period, the cutoff frequency of low-pass filter is 11 Hz, and the difference equation can be expressed as follows:

(1) $$\begin{array}{c} y\left(nT\right)=2y\left(nT-T\right)-y\left(nT-2T\right)-2x\left(nT-6T\right)+x\left(nT-12T\right)+x\left(nT\right). \end{array}$$

The cutoff frequency of the high-pass filter is 2 Hz, and the difference equation can be expressed as

(2) $$\begin{array}{c} y\left(nT\right)=y\left(nT-T\right)-x\left(nT\right)+32x\left(nT-16T\right)+x\left(nT-32T\right). \end{array}$$

*(2) Amplification*. R wave in the QRS wave group is the steepest wave in an ECG signal cycle. In order to distinguish QRS waves from other ECG signals conveniently, the corresponding differential method is needed to amplify the steep slope characteristics of QRS wave groups. The specific difference equation is as follows:

(3) $$\begin{array}{c} y\left(nT\right)=x\left(nT\right)-x\left(xT-2T\right). \end{array}$$

The high-frequency characteristics can be enhanced by a nonlinear square function, whose equation can be expressed as

(4) $$\begin{array}{c} y\left(nT\right)={\left[x\left(nT\right)\right]}^{2}. \end{array}$$

*(3) Threshold Dynamic Adjustment and Search*. Threshold dynamic adjustment and search belong to the core part of the algorithm, through which to search the peak value of ECG signal, through a certain equation to update the threshold, and combined with backtracking detection, bidirectional discrimination, and other content to detect. The process of this method is complex, which has been described in detail in paper [7]. Using the method provided by it, the final detection can be completed.

The article "Electrocardiogram Signal Classification in the Diagnosis of Heart Disease Based on RBF Neural Network" was published in 2022. Journal: Comput Math Methods Med.

### 2.2. Data Preprocessing

#### 2.2.1. Pretreatment Basis

*K*-means clustering method is also called the *K*-means clustering algorithm. Firstly, the sample objects are randomly selected, then the selected objects are regarded as the center of the clustering process, and then other object samples are also put into the model to calculate the distance between each object sample and the cluster center sample selected randomly. The nearest center sample will assign it to. When the condition that the object is fully allocated is satisfied, it is recalculated. The process is repeated to meet the conditions and stop the computation. The termination condition of this paper is the minimum center change, that is, the number of cluster center changes is the smallest, and the clustering is stopped.

There is no best method for *K* value in theory. Only when clustering, we try to make manual selection repeatedly. But in the process of this step, *K* is taken as 2 to screen the corresponding segments of these clusters.

Based on the results of feature extraction, this paper will adopt the interception-clustering filtering method [16] for sample preprocessing.

#### 2.2.2. Truncation Process

In the above, the QRS wave group of samples has been extracted with high accuracy, so according to the information of extracted feature points, samples can be effectively truncated for subsequent clustering screening, so as to improve the accuracy of classification results (Figure 3).

Normally, the heartbeat of normal people is the lowest once a second and the highest is twice a second. The corresponding heartbeat time of the heart rate is its corresponding ECG cycle. The converted range is about 600 ms to 1000 ms. The equation is as follows.

(5) $$\begin{array}{c} T=\frac{r}{t_{h}}, \end{array}$$

where *T* is the period corresponding to ECG, *R* is the heart rate, and *t*_*h*_ is the number of heartbeats in the corresponding time of heart rate.

Let R wave correspond to *R*_*i*_, Q wave correspond to *Q*_*i*_, and S wave correspond to *S*_*i*_, where *i* = 1, 2, 3, 4 ⋯ *N*, *N* is the total set of R waves in the sample.

(6) $$\begin{array}{c} \left\{\begin{array}{c} \begin{array}{c} Q_{i}-Q_{i-1}=T\;\left(i\neq 0\right),\\ Q_{i+1}-Q_{i}=T\;\left(i\neq N\right),\\ Q_{i+1}-Q_{i}=T\;\left(i\neq N\right), \end{array}\\ R_{i}-R_{i-1}=T\;\left(i\neq 0\right),\\ R_{i+1}-R_{i}=T\;\left(i\neq N\right),\\ S_{i}-S_{i-1}=T\;\left(i\neq 0\right),\\ S_{i+1}-S_{i}=T\;\left(i\neq N\right). \end{array}\right. \end{array}$$

If the corresponding time limit of the QRS wave group is *t*_QRS*i*_ with units in milliseconds, it can be inferred.

(7) $$\begin{array}{c} 60\leq t_{\text{QRS}i}\leq 100. \end{array}$$

Heart rate can be effectively detected by T wave and QRS wave group. Let T wave correspond to *T*_*i*_, where *i* = 1, 2, 3, 4, ⋯, *N*, *N* is the total set of R waves in the sample.

(8) $$\begin{array}{c} r_{t}=T_{i}-Q_{i}. \end{array}$$

The feature extraction has been carried out above, and the experimental data are analyzed. The *R*_*i*_ + 500 ms corresponding to R wave are truncated separately and saved as truncated samples, which will be used for the next clustering analysis. The data content stored in each row corresponds to an interval intercepted in this paper.

The article "Electrocardiogram Signal Classification in the Diagnosis of Heart Disease Based on RBF Neural Network" was published in 2022. Journal: Comput Math Methods Med.

#### 2.2.3. Screening Process

Suppose the input sample is *S* = *x*_1_, *x*_2_, ⋯, *x*_*m*_ and *m* are the width of the cut sample, and the centers of the initial *K* samples are set to *μ*_1_, ⋯, *μ*_*K*_, respectively. For any sample *x*_*i*_(*i* = 1, 2, ⋯, *m*), according to the Euclidean distance equation, the nearest class of the center can be computed. Let *D* be the width of the truncated sample. The equation is as follows:

(9) $$\begin{array}{c} \text{dist}\left(x_{i},x_{j}\right)=\sqrt{\overset{D}{\underset{d=1}{\sum }}{\left(x_{i}d-x_{j}d\right)}^{2}}. \end{array}$$

In the process of continuous iteration, we need to substitute a condition to stop iteration. As mentioned above, the method of error sum and criterion function is adopted to stop iteration. The function model is as follows:

(10) $$\begin{array}{c} J=\overset{K}{\underset{k=1}{\sum }}\underset{x_{i}\epsilon C_{k}}{\sum }\text{d}\text{ist}\left(x_{i},{Ce}_{k}\right). \end{array}$$

When the value of △*J* is less than the threshold set, the iteration stops.

In the case of this experiment, the number of samples in the cluster corresponding to the normal class is much larger than that of the abnormal cluster, so the abnormal data is eliminated directly. The screening process has been completed.

### 2.3. Feature Selection

#### 2.3.1. Selection Process

Assuming that the number of data bars is *n* and the dimension is *d*, the method can be summarized as follows:

1. The filtered data are composed of *d* rows and *n* column matrix *M*′
2. Subtract all rows of *M*′ from the average of the row
3. Calculate the covariance matrix *M*′ and the required value
4. Arrange the eigenvectors
5. Constituting a new matrix *P*, the matrix *P* is the result of reducing the dimension

For the covariance matrix, the sample size is assumed to be *n*, the average is *X*, the standard deviation is *s*, and the variance is *s*^2^. The details are as follows:

(11) $$\begin{array}{c} \bar{X}=\frac{\sum_{i=1}^{n}X_{i}}{n}, \end{array}$$

(12) $$\begin{array}{c} \;s=\sqrt{\frac{\sum_{i=1}^{n}{\left(X_{i}-\bar{X}\right)}^{2}}{n-1}}. \end{array}$$

(13) $$\begin{array}{c} \;s^{2}=\frac{\sum_{i=1}^{n}{\left(X_{i}-\bar{X}\right)}^{2}}{n-1}. \end{array}$$

By computing the correlation by covariance, the following definitions are given:

(14) $$\begin{array}{c} \mathrm{cov}\left(X,Y\right)=\frac{\sum_{i=1}^{n}\left(X_{i}-\bar{X}\right)\left(Y_{i}-\bar{Y}\right)}{n-1}. \end{array}$$

In fact, this paper solves a problem with multiple dimensions, so it needs to calculate multiple covariances. To achieve this process, a matrix is needed to organize the data, so a covariance matrix is defined:

(15) $$\begin{array}{c} C_{n\times n}=\left(c_{i,j},c_{i,j}=\mathrm{cov}\left({\text{Dim}}_{i},{\text{Dim}}_{j}\right)\right). \end{array}$$

Covariance matrix can be used:

(16) $$\begin{array}{c} M^{\prime }=\left(\begin{array}{ccc} \mathrm{cov}\left(x,x\right) & \mathrm{cov}\left(x,y\right) & \mathrm{cov}\left(x,z\right)\\ \mathrm{cov}\left(y,x\right) & \mathrm{cov}\left(y,y\right) & \mathrm{cov}\left(y,z\right)\\ \mathrm{cov}\left(z,x\right) & \mathrm{cov}\left(z,y\right) & \mathrm{cov}\left(z,z\right) \end{array}\right). \end{array}$$

Then, the eigenvalues and eigenvectors are calculated according to the actual situation to complete the corresponding operation of dimensionality reduction.

The article "Electrocardiogram Signal Classification in the Diagnosis of Heart Disease Based on RBF Neural Network" was published in 2022. Journal: Comput Math Methods Med.

### 2.4. Classifier Design

#### 2.4.1. Method Selection

The supervised classifier based on RBF neural network is adopted in this paper. Compared with the traditional BF method, it has the advantages of fast learning, strong autonomy, linear output, and good classification effect [17]. Therefore, this method is chosen as the implemented classifier in this paper.

#### 2.4.2. Implementation Process

In general, the Euclidean distance between any point in space and another point, i.e., the distance between *x* and  *x*_*c*_, is recorded as a monotone equation:

(17) $$\begin{array}{c} k\left(\left|x-x_{c}\right|\right). \end{array}$$

The function commonly used in the model is Gauss Radial Basis Kernel Function [3], which can be expressed in the form of

(18) $$\begin{array}{c} k\left(\left|x-x_{c}\right|\right)=\exp\left\{\frac{-{\left|\left|x-x_{c}\right|\right|}^{2}}{2\sigma^{2}}\right\}. \end{array}$$

In the above equations,  *x*_*c*_ is defined as the midpoint of the kernel function and *σ* is the parameter of the width of the function, which is used to control the range of the function.

RBF neural network is actually a hierarchical structure, which includes three parts: input, hiding, and output. The transformation from input to hidden level is nonlinear, while the change from hidden to output level is linear. The output layer sums and outputs the output weights of the hidden layer. Let *n* be the total number of samples, and the given training sample is expressed as

(19) $$\begin{array}{c} X_{n}=\left\{x_{n1},x_{n2},\cdots ,x_{n,m-1},x_{nm}\right\},\left(n=1,2,\cdots ,N\right). \end{array}$$

The output after learning is defined as

(20) $$\begin{array}{c} Y_{n}\left(n=1,2,\cdots ,N\right). \end{array}$$

The base function is defined as *φ*(*x*, *x*_*i*_) above. The output of the base function is expressed as the output corresponding to the hidden unit *i*, and the corresponding center point of the base function can be expressed as

(21) $$\begin{array}{c} i_{n}=\left\{i_{n1},i_{n2},\cdots ,i_{n,m-1},i_{\text{n}m}\right\},\left(n=1,2,\cdots ,N\right). \end{array}$$

We set the initial value:

(22) $$\begin{array}{c} c_{jn}=\min n+\frac{\max N-\min\;N}{2n}+\left(j-1\right)\frac{\max N-N}{n},\left(j=1,2,\cdots ,n\right). \end{array}$$

The corresponding width is defined as

(23) $$\begin{array}{c} d_{n}\left(n=1,2,\cdots ,N\right). \end{array}$$

The calculation method of width can be expressed as

(24) $$\begin{array}{c} d_{n}=\sqrt{\frac{1}{N}\overset{N}{\underset{k=1}{\sum }}\left(x_{n}^{k}-c_{jn}\right)}. \end{array}$$

The corresponding weight can be expressed as

(25) $$\begin{array}{c} \omega_{n}\left(n=1,2,\cdots ,N\right). \end{array}$$

The overall structure of the neural network is shown in Figure 4.

The article "Electrocardiogram Signal Classification in the Diagnosis of Heart Disease Based on RBF Neural Network" was published in 2022. Journal: Comput Math Methods Med.

To sum up, the following summaries can be made:

(1) Initialization of parameters: according to Equation (20), the iteration *ε* jump-out accuracy is given
(2) When the output is generated, the RMS value of root mean square error is calculated. *O*_*k*_ represents the vector of expected output. The RMS equation is as follows:
  (26) $$\begin{array}{c} \text{RMS}=\sqrt{\frac{\sum_{i=1}^{N}\sum_{k=1}^{n}\left(O_{k}-Y_{k}\right)}{nN}.} \end{array}$$
 When RMS ≤ *ε*, the training is completed and the model is generated. Instead, it uses Equation (3)
(3) The adjustment parameters are recalculated and output; skip to Equation (2)

## 3. Experimental Method

### 3.1. Implementation Process

#### 3.1.1. Brief Description

The implementation process of this paper can be summarized as follows. The flowchart is shown in Figure 5.

1. Input the sample model group and extract the feature by using the algorithm of paper [7]
2. All samples are processed into truncated samples according to their characteristics
3. Cluster analysis, eliminating abnormal truncated samples
4. Dimension reduction and feature selection
5. Classifier training and testing after training
6. Classification and evaluation are obtained through analysis

#### 3.1.2. Flowchart

### 3.2. Experimental Process

#### 3.2.1. Description

When the training is completed, the classification of ECG signals using this method can be summarized as follows. The flowchart is shown in Figure 6 and detailed as follows:

1. Input the sample model group and extract the feature by using the algorithm of paper [7]
2. Samples are processed into truncated samples according to their characteristics
3. Cluster analysis, eliminating abnormal truncated samples
4. Dimension reduction and feature selection
5. Classifier is used to classify score, and the output is normal when the threshold is reached; otherwise, it is abnormal

The article "Electrocardiogram Signal Classification in the Diagnosis of Heart Disease Based on RBF Neural Network" was published in 2022. Journal: Comput Math Methods Med.

#### 3.2.2. Schematic Diagram

## 4. Results

### 4.1. Data Sources

The experimental data in this paper are from the MIT-BIH ECG database [18], which is provided by MIT and is often used to study arrhythmia and other heart symptoms. The files in the database are composed of three parts: the header file which stores the sampling rate and the length of the data, the data file which stores the ECG data in the binary format, and the annotation file which stores the detailed description. The most important value of the latter is the actual position of each wave in the data file, which can be used to check the reliability of feature extraction. The corresponding feature extraction algorithm [7] that was previously proposed is relatively mature, and its reliability can reach 99.3%. Even if there is abnormal feature extraction content, it can be basically eliminated through the above screening process, so there is no more excessive research on reliability.

### 4.2. Classification Criteria

As for the classification of ECG signals, the American Association for the Advancement of Medical Instruments (AAMI) has drawn up the relevant rule paper [19], which classifies ECG [20] beats into normal N-type, supraventricular abnormal signal S-type, abnormal signal V-type caused by ventricular abnormalities, F-type, fusion signal, which may contain a variety of abnormalities, and Q-type, which cannot be classified. Type U refers to the unreadable type; in addition, there are U, X, O types which do not belong to the category of ECG signals. In summary, in fact, except for the N-type, which includes the normal ECG signal type, the other basic types belong to the abnormal category. Therefore, the core of classification of ECG is how to distinguish the normal ECG signal accurately.

### 4.3. Experimental Results

#### 4.3.1. First Experiment

In this paper, 8000 sample models are used to identify abnormal ECG signals, including the above-mentioned situations, of which 5000 are used for training and 3000 for testing. The confusion matrix is shown in Table 1.

The results show that the accuracy of normal ECG signal detection can reach *99.71%*, abnormal ECG signal detection can reach *97.50%*, and comprehensive accuracy can reach *98.77%*.

The article "Electrocardiogram Signal Classification in the Diagnosis of Heart Disease Based on RBF Neural Network" was published in 2022. Journal: Comput Math Methods Med.

#### 4.3.2. Crossover Experiment

In order to verify the accuracy of the method, this paper subsequently carried out cross-validation [21] of the method. In the form of cross-validation, this paper selected 10-fold cross-validation, 5-fold cross-validation, and 2-fold cross-validation, respectively. There are two main reasons for conducting crossover experiments; one is to verify the accuracy, and the other is to study the influence of training quantity on test results.

According to the ideal state, the more training samples, the higher the final classification accuracy of the training model, and the limited number of actual samples; and because the interference of other factors does not necessarily meet the final results of this theory, this paper is only used for the accuracy of detection methods for crossover experiments.

Firstly, a 2-fold crossover experiment was conducted. For 8000 samples, 4000 samples were used for training and 4000 samples were used for testing. The results show that the accuracy of normal ECG signal detection can reach *99.96%*, abnormal ECG signal detection can reach *96.76%*, and comprehensive accuracy can reach 98.70%. The confusion matrix of the classification results is shown in Table 2.

Subsequently, 5-fold crossover experiment was carried out. For 8000 samples, 6400 samples were used for training and 1600 samples were used for testing. The results show that the accuracy of normal ECG signal detection can reach *99.79%*, abnormal ECG signal detection can reach *97.89%*, and comprehensive accuracy can reach 99.00%. The confusion matrix is shown in Table 3.

Finally, a 10-fold crossover experiment was conducted. For 8000 samples, 7200 samples were used for training and 800 samples for testing. The results show that the accuracy of normal ECG signal detection can reach *99.78%*, abnormal ECG signal detection can reach *97.61%*, and comprehensive accuracy can reach 98.88%. The confusion matrix [22] is shown in Table 4.

#### 4.3.3. Comparative Experimental Evaluation

In the comparative experiment, the technology is replaced by other methods in the feature extraction stage and classifier selection stage, and the cross experiments are carried out, respectively.

In the stage of feature extraction, wavelet transform method and neural network extraction method [23] are used to replace them, while in the stage of classifier selection BF neural network method is used to replace them. The method used in this paper does not optimize it, only using the corresponding algorithm provided by other people in the network resources to carry out relevant comparative experiments. From this, we can get the replacement method as shown in Table 5.

The article "Electrocardiogram Signal Classification in the Diagnosis of Heart Disease Based on RBF Neural Network" was published in 2022. Journal: Comput Math Methods Med.

It can be seen that besides using wavelet transform in the process of feature extraction, the accuracy of other methods is different from that of the methods proposed in this paper.

## 5. Discussion

In this paper, the classification of ECG signals is implemented by machine learning [24]. Firstly, the feature extraction is carried out according to the relevant methods provided in Section 2.1 of this paper. Then, according to the result of feature extraction, the samples are truncated, the samples are clustered and analyzed, some special truncated samples are eliminated, and the process of data prepossessing is completed. After the screening, the sample features are selected and the PCA is used. A method is used to reduce the dimension; and the first training of the classifier is carried out afterwards. Next, three cross experiments of 2-fold, 5-fold, and 10-fold are carried out, and the results are good. Finally, some methods in the process are replaced by comparative experiments, and finally, the corresponding methods in this paper are realized.

This paper focuses on the supplement to this field, which is also the innovation of this paper. Although there are a variety of corresponding technical methods in the research literature in this field, with the upgrading and development of information technology, it is inevitable to supplement many contents in this field, so the research content of this paper is of great significance.

## 6. Conclusion

According to the comprehensive test results, the detection accuracy of normal ECG signals can reach *99.74%*, the detection of abnormal ECG signals can reach 97.53%, and the comprehensive accuracy rate can reach *98.98%*. Although there is room for improvement in the detection of abnormal ECG signals, this does not affect the good classification effect that this method can show in the classification study of ECG signals. However, the recognition accuracy of abnormal ECG signals can still continue to be improved, and we will further study this in the future.

The following research direction of this paper is to develop the entity system through the above methods and consider combining it into telemedicine-related technology and mobile medical technology. Secondly, the methods used in the research process will still optimize the parameters [25]. When new and better technical heart diagnostics techniques appear, the new methods will be incorporated into or applied to the existing approach in the future. The current type of approach in our paper has strong clinical potential in cardiac diagnosis and treatment.

The article "Electrocardiogram Signal Classification in the Diagnosis of Heart Disease Based on RBF Neural Network" was published in 2022. Journal: Comput Math Methods Med.

## Figures and Tables

**Figure 1:** A schematic diagram of one or two human leads in registering ECG signals.

**Figure 2:** Schematic diagram of an ECG cycle.

**Figure 3:** Examples of the same sample truncation results in the QRS wave group.

**Figure 4:** Supervised classifier based on RBF neural network for classification of ECG signals at different cycles.

**Figure 5:** Procedural flowchart of method implementation.

**Figure 6:** Procedural flowchart of our method.

**Table 1:** Confusion matrix for initial experimental results.

		Prediction		
		Normal	Abnormal	Total
Actual	Normal	1716	5	1721
	Abnormal	32	1247	1279
	Total	1748	1252	3000

**Table 2:** Twofold confusion matrix for cross-experimental results.

		Prediction		
		Normal	Abnormal	Total
Actual	Normal	2425	1	2426
	Abnormal	51	1523	1574
	Total	2476	1524	4000

**Table 3:** Fivefold confusion matrix for crossover experimental results.

		Prediction		
		Normal	Abnormal	Total
Actual	Normal	934	2	936
	Abnormal	14	650	664
	Total	948	652	1600

**Table 4:** 10-fold confusion matrix for crossover experimental results.

		Prediction		
		Normal	Abnormal	Total
Actual	Normal	464	1	465
	Abnormal	8	327	335
	Total	471	329	800

**Table 5:** Method replacement consolidation table.

Substitution selection	Our method	BF neural network
The method in this paper	Method 1	Method 4
Wavelet transform	Method 2	Method 5
BF neural network	Method 3	Method 6

## Data Availability

The experimental data in this paper are from the MIT-BIH ECG database.
